# A novel approach for automatic segmentation of prostate and its lesion regions on magnetic resonance imaging

**DOI:** 10.3389/fonc.2023.1095353

**Published:** 2023-04-19

**Authors:** Huipeng Ren, Chengjuan Ren, Ziyu Guo, Guangnan Zhang, Xiaohui Luo, Zhuanqin Ren, Hongzhe Tian, Wei Li, Hao Yuan, Lele Hao, Jiacheng Wang, Ming Zhang

**Affiliations:** ^1^Department of Medical Imaging, First Affiliated Hospital of Xi’an Jiaotong University, Xi’an, China; ^2^Department of Medical Imaging, Baoji Central Hospital, Baoji, China; ^3^Department of Language Intelligence, Sichuan International Studies University, Chongqing, China; ^4^Department of Computer Science & Engineering, The Chinese University of Hong Kong, Hong Kong, Hong Kong SAR, China; ^5^Department of Computer Science, Baoji University of Arts and Sciences, Baoji, China; ^6^Department of Urology, Baoji Central Hospital, Baoji, China

**Keywords:** prostate cancer, convolution neural network, dense block, attention mechanism, U-Net

## Abstract

**Objective:**

To develop an accurate and automatic segmentation model based on convolution neural network to segment the prostate and its lesion regions.

**Methods:**

Of all 180 subjects, 122 healthy individuals and 58 patients with prostate cancer were included. For each subject, all slices of the prostate were comprised in the DWIs. A novel DCNN is proposed to automatically segment the prostate and its lesion regions. This model is inspired by the U-Net model with the encoding-decoding path as the backbone, importing dense block, attention mechanism techniques, and group norm-Atrous Spatial Pyramidal Pooling. Data augmentation was used to avoid overfitting in training. In the experimental phase, the data set was randomly divided into a training (70%), testing set (30%). four-fold cross-validation methods were used to obtain results for each metric.

**Results:**

The proposed model achieved in terms of Iou, Dice score, accuracy, sensitivity, 95% Hausdorff Distance, 86.82%,93.90%, 94.11%, 93.8%,7.84 for the prostate, 79.2%, 89.51%, 88.43%,89.31%,8.39 for lesion region in segmentation. Compared to the state-of-the-art models, FCN, U-Net, U-Net++, and ResU-Net, the segmentation model achieved more promising results.

**Conclusion:**

The proposed model yielded excellent performance in accurate and automatic segmentation of the prostate and lesion regions, revealing that the novel deep convolutional neural network could be used in clinical disease treatment and diagnosis.

## Introduction

Prostate cancer (PCa) is a significantly prevalent cancer among men, accounting for a half about of cancer diagnoses and the fifth highest cause of mortality (1). The age at which prostate cancer typically appears is relatively late, with most cases occurring after the age of 55, and the incidence gradually increases thereafter, peaking between the ages of 70 and 80. However, in cases of familial hereditary prostate cancer, the age of onset tends to be slightly earlier, with 43% of affected individuals developing the disease before the age of 55 (2). Prostate cancer can be diagnosed, treated, and monitored using several imaging modalities, including transrectal ultrasound (TRUS), magnetic resonance imaging (MRI), and computed tomography (CT). These imaging techniques are commonly used in clinical practice to aid in the diagnosis and management of prostate cancer.

In recent years, MRI technology has advanced significantly, providing high-level spatial resolution and soft tissue conspicuity, which makes MRI a suitable imaging technique for prostate segmentaion, staging and volum calculation of prostate cancer. The high-level spatial resolution and soft tissue conspicuity of MRI make it appropriate for prostate segmentation, staging and volume calculation of prostate cancer (3). In the same way, dynamic contrast-enhanced MRI (DCE-MRI) can be used to recognize malignant structures according to the spread rate of contrast agents (4–6), and magnetic resonance spectroscopy can discriminate malignant tissues in terms of the relative intensities of different metabolites (e.g., citric acid, choline, and creatine).

Traditional segmentation approaches of prostate or lesion area include contour and shape-based approaches and region-based techniques, and some hybrid methods. The prostate edge or boundary is applied to prostate segmentation. For example, Zwiggelaar et al. (7) employed a system of first and second-order Lindeberg directional derivatives (8) coordinates in polar coordinates to discern edges. To obtain the prostate boundary, the inverse shift of the longest curve was chosen after non-extreme on the disconnected curve in the vertical dimension. Flores-Tapia et al. (9) traced the boundary using *a priori* form information of the prostate by shifting a little filter mask over a feature space that was constructed from the Haar wavelet in the multiresolution structure. Klein et al. (10) adopted a multi-atlas method to segment the prostate. The training data was aligned to with the test data by affine alignment and subsequent non-rigid alignment with three b-spline bars in the framework. Gao et al. (11) developed the training set shape as a point cloud. The shape prior and local image statistics were integrated into the energy function to minimize the energy function for prostate segmentation in a level-set format. Manual segmentation remains the most widely utilized method for achieving accurate segmentation of the prostate and lesion region. it is not only a very time-consuming task and is subject to tissue variations. Additionally, it also heavily depends on the level of manual expertise and experience, which can lead to low reproducibility and higher observer variation.

In order to overcome those issues, there is an urgent need for reliable automatic segmentation of the prostate and lesion region in daily clinical practice. In 2012, Hilton’s team participated in the ImageNet image recognition competition for the first time. AlexNet (12) was awarded the championship and crushed the second classification performance of support vector machine. As a result, the development of deep learning technology was advancing by leaps and bounds, and it was applied in many directions. CNN continuously extracts features from all layers, from local to overall features. CNNs are obtaining a concern in the medical image field due to the state-of-the-art scores on plentiful image identification and segmentation tasks. One of the outstanding representative works is that Ronneberger et al. (13) proposed the U-Net model and made full use of the limited and valuable training set to boost segmentation performance. The U-shaped structure makes the localization accurate for medical images instead of simple binary classification. The overall process of U-Net includes encoding and decoding, with only a convolutional layer and no fully connected layer. Currently, U-Net is arguably an even hotter segmentation network. Lai et al. (14) proposed a network for automatic segmentation for prostate zone and cancer RoI by Segnet. They considered different sequences into three channels of an image and used PROSTATEx dataset to train the network. At last, the T2W + DWI + ADC scheme obtained the best grade with a Dice similarity coefficient of 90.45%. Wang et al. (15) presented a 3D CNN model and used the attention mechanism to fully mining more useful features encoded in the network for prostate segmentation. To enhance local prostate cancer control, Chen et al. (16) proposed three-branch U-Net to distinguish different targets for segmentation in MRI. Deep monitoring policies were combined into the network to accelerate convergence and boost network capabilities. To reduce the loss of structural and spatial information, Orlando et al. (17) designed a 3D segmentation model based on 2D U-Net for the prostate. The novel model can offer a quick and effective segmentation compared to other methods.

It is very challenging to get an automatic segmentation model with high performance for the prostate and its lesion region. The ambiguity of each tissue boundary inside the image makes it difficult to distinguish it from the heterogeneous tissue within the surrounding prostate, further resulting in under-segmentation or over-segmentation. Additionally, the varying sizes and shapes of prostate glands among individuals pose challenges in modeling pervasive learning. The above reasons make regional resection of prostate cancer difficult and challenging. To address these challenges, we propose a new network for the automatic segmentation of prostate and prostate cancer regions. Our network is inspired by U-Net and utilizes a simple but effective attention module, which could be broadly used to improve the capability of CNN. In short, the attention network is in charge of focusing attention on certain important features of an image which improves the segmentation quality. Dense block also is employed to mitigate gradient disappearance and enhance the propagation of features in the model. Additionally, the dense block is employed to mitigate gradient disappearance and enhance the propagation of features, resulting in more abstracted interested features. In the data preparation phase, data augmentation is utilized to solve the problem of overfitting the model due to limited amount of date. The main contributions of this work are as follows.

Firstly, to fulfill the pixel-wise segmentation, a novel CNN model is proposed in this study. The model uses lengthy skip connections between the relative stages of the encoder and decoder and facilitates end-to-end training. To expand the perceptual field of the convolution kernel without loss of resolution (no down-sampling), group norm- Atrous Spatial Pyramidal Pooling is introduced in our model.

Secondly, to stabilize parameter updating and keep a more effective image feature, the dense block is incorporated to utilize short skip connections between different convolutional layers.

Thirdly, the introduction of CBAM is used to make the network more seneitive to the characteristics of both channel and space dimensions. In this study, CBAM allows the model to focus more features on the prostate and its lesion areas from space and channels. Thus, the model helps the flow of information within the network by learning which information should be emphasized and suppressed.

Finally, we evaluate the proposed model on a real dataset and show its effectiveness by outperforming state-of-the-art segmentation models on multiple evaluation indices.

## Materials and methods

### Datasets

The data were conducted with MRI from 180 patients (122 healthy individuals and 58 patients with prostate cancer from pathology report). Data were acquired using the GE3.0T 750 MR between January 2018 and May 2021. Informed consent was obtained from all patients. The input sequence was the DWI format. DWI: TE82ms, TR 6000ms, Thickness 3.5 mm, Scan Matrix 128 ×128, b value 0, 500, 1000, 1500mm^2^/s. To ensure that the ground truth segmentation was as correct as possible, six experienced prostate clinicians participated in analyzing and annotating the prostate MR images. Three clinicians spent 3 months demarcating all masks with the monitoring interface (Labelme). To compensate for inaccurate label borders that may be caused by subjective physician judgment. The other three experts reviewed and revised the annotating masks. The overlapping part of the two outlined areas was finally considered as the labeled target.

### Data pre-processing

The primary pre-processing stages used in this approach are data enhancement and image normalization. Data augmentation is used to address overfitting issues in the raw data. It involves following operations: image rotation by a variable number of degrees (-10, 0, 45,60); shifting the image up, down, left, and right; and resizing the image 0.9 and 1.1 times. Finally, the number of prostate and lesion region samples is 1936 and 514. Deep learning models are required to normalize their input data to ensure an adequate convergence point. Normalization can be achieved using different strategies, such as min-max norm and the linear function which converts the input data to the range [0, 1]. This operation achieves equal scaling of the original images. Another approach is 0-mean normalization, which normalizes the raw data set to have a mean of 0 and a variance of 1. In this study, we use a mini–maxi norm to apply the linear transformation to the raw data range. The formula is Xnorm=(X- Xmin)/(Xmax- Xmin), where Xnorm is the normalized data, X is the raw data, and Xmax and Xmin are the maximum and minimum values of the raw data set, respectively. This unique technique is suitable for the image at a predefined mask. The data normalization procedure is performed on the test data to obtain homogeneity, as necessary for the model to provide robust results.

### The proposed model

The model is encouraged by the classical U-Net network (13) and considered the decoding-encoding idea. Meantime, the model introduces dense blocks, convolution block attention module (CBAM) and group norm-Atrous Spatial Pyramidal Pooling (GN-ASPP) (18) to capture more feature representation in segmentation. To effectively utilize shallow information, the proposed model fuses features from the contraction path into the expansion path at both symmetrical and asymmetrical levels. **Figure 1** presents the details of the proposed model. DWI image is considered for model input. The convolution operations inside the model are all performed using 3×3 marked in red. The model consists of a contraction path (left side) and an expansion path (right side). The contraction path is designed to produce contextual information and the extension path is for precise positioning, and the two paths are mutually synchronous. The whole architecture utilizes short skip connections between various convolution layers at each step, which assists in steady parameter optimization. The union of long and short skips boosts the general efficiency of the network (19). The contraction path is responsible for downsampling and the number of channels increases from 64 to 1024. In the expansive path, each step involves an up-convolution of the prostate feature map, followed by a 2×2 convolution operation that reduces the number of feature channels by half. Another component is a concatenation with the tailoring prostate feature from the contracting path of the same layer. Apart from that, two 3×3 convolutions, each postulated with a ReLU and a CBAM, are included in the expansive path. The last layer employs three convolutions and a spatial pyramidal pooling with rates (6, 12, 18) to determine the number of classes. As boundary pixels are lost on each convolution, trimming is necessary.

**Figure 1:** Structure of the proposed method. Yellow for CBMA module, dark blue for dense unit, with ASSP added to the end of the model.

A dense block (20) is a dense concatenation of numerous composite functions which makes up batch normalization, ReLU layer, convolutional layer, and dropout layer. It serves to mitigate the gradient disappearance and enhance the propagation of the prostate and its lesion features and reuse them in the subsequent network layer. The CBAM module (21) uses the attention mechanism to optionally optimize the multi-dimension image features and extract the interest features at each layer, inhibiting more non-relative noise. The network can generate the channel and spatial attention map by separately mining the inter-channel and inter-spatial relationship of features, which explains ‘what’ and ‘where’ issues. CBAM structure is made up of channel attention and spatial attention. The input DWI map is F (2-channel). It is also an intermediate feature map. CBAM defines a 1D channel attention map M_C_ and 1D spatial attention map M_S_ (18).


$$\begin{array}{l} M_{C}\left(F\right)=\sigma \left(MLP\left(AvgPool\left(F\right)\right)+MLP\left(MaxPool\left(F\right)\right)\right)\\ =\text{σ}\left(W_{1}\left(W_{0}\left(F_{avg}^{C}\right)\right)+W_{1}\left(W_{0}\left(F_{max}^{C}\right)\right)\right) \end{array}$$

Where σ is the sigmoid function, W_0_∈R^(c/r×c)^, and W_1_∈R^(c/r×c)^. r denotes the reduction ratio. The hidden activation size is set to R ^C/r×1×1^. Note that multi-layer (MLP) weights, W_0_ and W_1_, are shared for both inputs and the ReLU is followed by W_0_. $F_{avg}^{C}$ and $F_{max}^{C}$ denote two spatial context descriptors.

Where f^(7*7)^ represents a convolution operation with a filter size of 7*7.

The attention principle can be explained as follows:

F’=M_C_ (F)⊗F
F’’=M_S_ (F’) ⊗F’

⊗ representatives element-wise multiplication. F^’’ denotes the final output.

The multi-scale feature maps obtained are then not directly used to predict the condition of object regions. To achieve more precise performance of the prostate and its lesion regions, we employ the spatial pyramidal pooling module to rescale attention features at various scales. As shown in **Figure 2**, features from up-sampling and dense block connections are fused to form a feature map of interest. The feature map is then processed by applying four parallel convolutions with different rates to collect various information. Our ASPP includes a 1×1 convolution and a triple 3×3 dilated convolution with rates of (6, 12, 18). Each convolution is followed by a normalization. We selected group norm (GN) over batch normalization because GN’s accuracy is fairly stable over a wide range of batch sizes.

**Figure 2:** Schematic representation of the spatial pyramid set (ASPP) for dilated convolution and group norm (GN).

### Evaluation of the proposed model

We evaluated the developed network in comparison with other state-of-the-art segmentation networks, including FCN (22), U-Net (13), U-Net++ (23), ResU-Net (24). To ensure a fair comparison, these models were retrained to produce the best separation results. During the training period, the training cross-entropy loss is exploited. The optimized method employed is Adam as it converges faster. The model was trained 150 times for almost all architectures. Checkpoint and stopping methods were utilized to reduce computation time.

To quantitatively assess the segmentation, we utilized several indicators, including Dice Similarity Coefficient (Dice), IoU, sensitivity, accuracy, and Hausdorff Distance (HD). Dice was utilized to assess the likelihood of similarity between the segmented volume and the ground truth. Dice are utilized to assess the likelihood of similarity between the segmented volume and the ground truth. Accuracy and Iou were appraised from the perspective of voxel classification for segmentation. Hausdorff distance is a measure that describes the degree of similarity between two sets of points. The dataset was divided into training (70%), and testing set (30%) when each experiment was conducted in a randomized manner. Four-fold cross-validation method was used to obtain experimental results. All training data was randomly divided into 4 sets, 3 of which were used for training and the remaining one for validation. When this round was completed, 3 parts were randomly selected again to train the data. Finally, the optimal parameters was selected from loss evaluation.

## Results

### Comparison of the state-of-the-art algorithms

#### Loss vs Epoch

The training process was recorded, as shown in **Figures 3** and **4**. These two figures represent the effect of prostate area and lesion area vs epoch, respectively. Each epoch is one round of data re-iterations. The two figures show similar loss trends in the prostate and its lesion segmentation. The loss decreases from epoch 0 to 60. The model starts convergence from epoch 60. Although the ResUnet model exhibits a higher loss value compared to other models, all models exhibit similar convergence trends, and the model slowly converges as the number of training sessions increases.

**Figure 3:** Loss vs epoch of prostate area on training data.

**Figure 4:** Loss vs epoch of prostate lesion area on training data.

#### Iou vs epoch

Iou is the intersection of the predicted and true results. It is often used as a metric to assess how well a model is learning. The curve chart of Iou vs epoch for the proposed algorithm is given in **Figures 5** and **6**, respectively. From 0 to 60 epochs, Iou of our method is unstable and fluctuates. But, the proposed approach is capable of producing better Iou than the state-of-the-art segmentation methods when the model converges to fit. In particular, it can be seen that the Iou of our algorithm is significantly greater than the other algorithms in **Figure 5**, which demonstrates that our model has better segmentation performance.

**Figure 5:** Iou vs epoch of the prostate area on testing data.

**Figure 6:** Iou vs epoch of prostate lesion area on testing data.

The segmentation performance was computed for the prostate and its lesion area with four cross-validations. In **Table 1**, the proposed network achieved an average dice sorce, Iou, accuracy, sensitivity for the prostate of 93.90%, 86.82%, 94.11%, and 93.80%. Our algorithm outperformed U-Net, U-Net++, FCN, and ResU-Net in Dice metrics by 1.7, 1.4, 2.6, and 7.19 percentage points and in terms of sensitivity metrics by 1.55, 2.68, 1.9, 10.5 percentage points for the prostate segmentation. In **Table 2**, for the segmentation performance of the prostate lesion, the proposed network yielded better results in terms of Dice score of 89.51%, Iou of 79.20%, accuracy of 88.43%, sensitivity of 89.31%, and 95%HD of 8.39 compared with the other 4 models. These findings suggest that this algorithm has superior performance compared to other models.

**Table 1:** Segmentation performance of prostate area for five models.

Model	Dice	Iou	Accuracy	Sensitivity	95%HD(mm)
U-Net	92.20%	85.81%	93.0%	92.35%	8.94
U-Net++	92.50%	84.90%	93.6%	91.12%	8.89
FCN	91.30%	84.62%	92.4%	91.90%	8.71
ResU-Net	86.71%	76.01%	89.51%	83.30%	8.51
Proposed	93.90%	86.82%	94.11%	93.80%	7.84

**Table 2:** Segmentation performance of prostate lesion area for five models.

Model	Dice	Iou	Accuracy	Sensitivity	95%HD(mm)
U-Net	87.50%	77.91%	87.40%	88.53%	9.01
U-Net++	88.20%	77.45%	86.21%	87.56%	8.82
FCN	85.31%	75.06%	86.11%	85.03%	8.73
ResU-Net	81.21%	69.14%	86.30%	81.19%	8.66
Proposed	89.51%	79.20%	88.43%	89.31%	8.39

We did ablation experiments to verify the effect of each module on our model in **Table 3**. The dense block, CBMA, GN-ASPP were gradually increased on the backbone. In our dataset, the ablation experiment was implemented with identical model parameters, e.g. Adam, learning rate, model initialization, and loss function. This result shows that the guidance technology is reinforcing to each other. Our approach achieved the best performance and could learn more robust representation from dense block, CBMA, and GN-ASPP.

**Table 3:** Ablation experiments for the segmentation of the prostate and its lesion regions (√notes to introduce this technology in the model).

	Backbone (U-Net with feature fusion)					
Dense Block	√	√	√		√	
CBMA	√	√		√		√
GN-ASPP	√		√	√		
Dice of Prostate/Prostate lesion regions	93.90%/89.55%	93.00%/88.34%	91.24%/88.67%	89.71%/87.94%	88.86%/ 87.81%	88.67%/ 86.31%

### Visualization of segmentation effect

**Figure 7** presents schematic images of the segmentation results obtained from our model. From the test results, we randomly selected 4 samples for the presentation of the results. Our model accurately distinguished between the prostate areas and lesion areas, with the segmentation of the prostate region being more accurate compared to the lesion area. These findings are consistent with the results presented in **Table 1** and **2**. To show the effect of CBAM in our model, the visualization attention results of the final layer of the model for the prostate lesion region are given in **Figure 8**. The rose mask denotes the area of interest which is the prostate lesion region.

**Figure 7:** Segmentation performance of the proposed method in 4 different patients (row), and columns from left to right show input image, ground truth, and segmentation results of the proposed model. In the experiments, non-target regions were masked black to provide greater clarity. The lesion region is marked in yellow, while the prostate region in rose.

**Figure 8:** Visualization of the final layer of our model for prostate lesion region.

## Discussion

In this study, we propose a novel DL-based architecture that utilizes the dense block and CBAM, as well as the GN-ASPP module, to fully leverage the complementary information encoded in different layers of the model. Our proposed method is designed to improve the segmentation performance of the prostate and its lesion regions and aid clinical diagnosis. The segmentation output is obtained through an end-to-end approach. The model performance was evaluated on a real dataset. The experimental setup consisted of several aspects: observing the loss value and Iou change of each algorithm during training, quantitative comparison of the performance of each model, and visualization of model results. Finally, it was demonstrated that the proposed segmentation method outperformed the results of the state-of-the-art methods for segmentation of the prostate and lesion region. Specifically, the proposed method exhibited excellent results, especially for the lesion region, which is of great significance for clinical diagnosis and treatment.

Several studies demonstrates artifical intelligence is valid in urology works (25–27), especially using DCNN to segment the prostate or determine prostate cancer. Zhu et al. (28) designed a DCNN model to segment the prostate zone and outer contour. The model was derived from a cascade of two models. One model was responsible for segmenting the prostate region and one for segmenting the prostate zone. However, an end-to-end model, like the one proposed in our study, is more efficient in reducing training time and facilitating clinical diagnosis. Duran et al. (29) also developed a novel CNN model for PCa segmentation with an attention mechanism. This strategy is similar to our approach. Moreover, we used CBAM in the model which focused on both the spatial dimension and the channel dimension. It is essential to design a model that extracts as many effective features as possible to automatically and accurately segment the prostate and its lesion region.

Firstly, we adopt a symmetrical architecture inspired by the classical U-Net, with a contraction path and an expansion path, copy and concatenate connections in the same layer, as well as a fusion of features in different layers. There is also a fusion of features in different layers. The main idea of the architecture is to continuously perform deeper feature extraction of prostate image features using the systolic network and to supplement the images lost by the systolic network using the expansion network. At the same time, in order to make more efficient use of the underlying feature information, we fuse the lower-down sampling features into the up-sampling features of the upper layer.

Secondly, the dense block is added to the left side of the model to allow for effective retention and propagation of the prostate and its lesion features. Then, the introduction of the attention mechanism allows the model to focus on areas of the prostate and its lesion in both spatial and channel dimensions, as shown in **Figure 8**. The huge number of parameters of the DCNN model affects the prediction results. Dense block and CBAM are integrated into the model to enhance the performance of the segmentation model without increasing the burden on the backbone (20, 21). To expand the perceptual field of the convolution kernel without loss of resolution (no down-sampling), GN-ASPP is introduced in our model.

Thirdly, some deep models for prostate cancer discrimination take the combination of image sequences as input (14, 30, 31) or the models take multi-branch outputs (16, 28). The more complex the model, the more training examples it requires, leading to a higher risk of overfitting. In contrast, our model takes a single image input and produces one branch output while still achieving excellent results.

Moreover, our method has the same convergence effect as the classical U-Net because of the backbone of the model, as shown in **Figures 3** and **4**. Meantime, our model has also similar convergence rates and effects in both the prostate and lesion regions, which demonstrates that the model has generalization properties.

Some restrictions of our study are worth mentioning (1), In deep learning, the more the amount of data, the better the final result will be. But in this study, data for model training is scarce (2), The operation efficiency of this network could be improved. For each neighborhood, the network has to run once, and for the overlapping part of the neighborhood, the network performs repeated operations (3), Initialization of parameters has a great impact on model training. Compared to the random initialization of the model parameters we studied, an effective initialization is more beneficial for the convergence of the model. To ensure the success of clinical application, it is essential to devep a robust and generalizable model. In the future, we will continue to collect more images of the prostate and increase the size of training set. Additionally, the combined use of data from different formats of MRI can compensate for the deficiencies of single data and improve the segmentation performance of the prostate and lesion regions.

In conclusion, we have proposed a DCNN model with dense block, convolution block attention module, and group norm-Atrous Spatial Pyramid Pooling for the segmentation of the prostate and its lesion regions. Experiments showed that this automatic segmentation model had excellent scores, which supports its potential to assist prostate disease diagnosis and treatment in clinical medicine.

## Data availability statement

The original contributions presented in the study are included in the article/supplementary material. Further inquiries can be directed to the corresponding author.

## Author contributions

MZ contributed to the conception and design of the article. HR and ZG analyzed and wrote the manuscript. ZG, CR, GZ, XL, ZR, HT, WL, HY, LH, and JW revised the manuscript. All authors contributed to the article and approved the submitted version.
